# Neuroprotective Effect of Turmeric Extract in Combination with Its Essential Oil and Enhanced Brain Bioavailability in an Animal Model

**DOI:** 10.1155/2021/6645720

**Published:** 2021-01-26

**Authors:** David Banji, Otilia J. F. Banji, Kavati Srinivas

**Affiliations:** ^1^Pharmacy Practice Research Unit, Department of Clinical Pharmacy, College of Pharmacy, Jazan University, Saudi Arabia; ^2^Nalanda College of Pharmacy, Nalgonda, India

## Abstract

**Purpose:**

The study evaluated the neuroprotective effect and pharmacokinetic profile of turmeric extract and their metabolites in the blood and brain in an aluminum-induced neurotoxic animal model.

**Methods:**

Swiss albino mice received turmeric extract (TE), TE-essential oil combination (TE+EO) at doses of 25 and 50 mg/kg/day orally, vehicle (control), and a positive control group. Neurotoxicity was induced by injecting aluminum chloride (40 mg/kg/day, i.p.), and the effect of the intervention was studied for 45 days. The pharmacokinetic and behavioral biochemical markers of brain function and brain histopathological changes were evaluated.

**Results:**

The AUC 0-*t* showed a 30.1 and 54.2 times higher free curcumin concentration in plasma with 25 mg/kg and 50 mg/kg of TE+EO vs. TE, respectively. The concentration of free curcumin in the brain was 11.01 and 13.71-fold higher for 25 mg/kg and 50 mg/kg of TE+EO vs. TE, respectively. Aluminum impairs spatial learning and memory, which was significantly reversed with TE+EO by 28.6% (25 mg/kg) and 39.4% (50 mg/kg). In the elevated plus maze test, 44.8% (25 mg/kg) and 67.1% (50 mg/kg) improvements were observed. A significant reduction in aluminum-induced lipid peroxidation was observed. Also, the levels of glutathione, acetylcholinesterase, and catalase were improved with TE+EO. Damage to the hippocampal pyramidal cells was averted with TE+EO.

**Conclusion:**

The neuroprotective and antioxidant response confirms the benefits of TE+EO against aluminum-induced neurotoxicity. The presence of free curcumin and its metabolites in the brain and plasma establishes its improved bioavailability and tissue distribution. Therefore, the benefits of TE+EO could be harnessed in neurodegenerative diseases.

## 1. Introduction

Human exposure to aluminum (Al) occurs through the environment, diet, and occupation [1]. The major sources of contact are cookware, cosmetics, and pharmaceutical products. Aluminum can enter the systemic circulation through the gastrointestinal tract and lungs [2]. Daily, nearly 10 mg of Al is taken into the human body, and up to 1% of Al undergoes absorption. Aluminum readily traverses through the blood-brain barrier exerting a detrimental impact on the central nervous system [3]. Elevated concentrations of Al have been observed in the hippocampus, cortex, and corpus callosum [4]. Chronic use of Al actuates the neuroinflammatory process by elevating the levels of proinflammatory cytokines and raising the risk of neuronal damage [5]. Aluminum is implicated in the pathogenesis of several neurodegenerative disorders like Alzheimer's disease, Parkinson's disease, and multiple sclerosis [1].

The accumulation of Al in the brain increases with age and the duration of exposure [6]. High concentrations of Al increase amyloid aggregation and deposition, which is the main feature of Alzheimer's disease [3]. Iron metabolism is impaired by Al^3+^, leading to its accumulation in neurons, resulting in oxidative damage [7].

Maintaining brain health is the most important as exposure to neurotoxins is unavoidable in everyday life. Plant-derived supplements are gaining popularity for improving brain health as these natural products are safer than synthetic drugs and can combat age-related oxidative processes [8]. Turmeric has been used for centuries throughout Asia as a food additive and traditional herbal medicine. Epidemiological evidence supports a link between better cognitive function in elderly Asians and curry consumption with turmeric [9]. Curcumin is the major yellow polyphenol present in the rhizomes of turmeric (Curcuma longa). Studies indicate that curcumin binds redox-active metals and has neuroprotective potential [10]. However, the health benefits of curcumin are blunted by its low water solubility, rapid metabolism, and quick elimination [11]. Moreover, curcumin readily converts to hydrophilic metabolites which can hamper their absorption [12]. Several studies also report that curcumin does not readily cross the blood-brain barrier and needs to be combined with bioavailability enhancer such as piperine [13, 14].

The presence of curcumin in the blood does not guarantee curcumin delivery in the brain, which is critical to combat neurological disorders. Therefore, turmeric extract-essential oil combination has been utilized to assess the availability of curcumin in the brain. This study is unique as it assesses the efficacy, pharmacokinetics, and tissue distribution of turmeric extracts in the Al-induced neurotoxicity model. Also, the ability of turmeric extracts to circumvent oxidative damage and memory deficits was ascertained.

## 2. Materials and Methods

### 2.1. Materials

Rhizomes of turmeric (Curcuma longa L., Zingiberaceae) identified by a qualified botanist were extracted with ethyl acetate to obtain the turmeric oleoresin. Curcuminoids were crystallized from the oleoresin to obtain turmeric extract (TE), which contains 95% curcuminoids. The rhizomes were steam distilled to get turmeric essential oil, which was blended with TE to form turmeric extract and essential oil combination (TE+EO). Aluminum chloride (AlCl_3_) was obtained from Central Drug House, New Delhi, India. In the pharmacokinetic analysis, reference standards such as curcumin (98%, HWI pharma services GmbH, Germany), demethoxycurcumin and bisdemethoxycurcumin (95%, Sigma-Aldrich, USA), curcumin glucuronide (94.6%, TLC Pharmaceutical Standards Ltd., Canada), curcumin sulfate (87.1%, TLC Pharmaceutical Standards Ltd., Canada), hexahydrocurcumin (90%, Fluka Chemie, Switzerland), and tetrahydrocurcumin (95%, Fluka Chemie, Switzerland) were used. All chemicals used for the biochemical estimations were of analytical reagent grade.

### 2.2. Phytochemical Analysis

The characterization and quantification of curcuminoids were established using UPLC-MS/MS (Waters Acquity H class UPLCMS/MS TQD system). An ambient BEH (Ethylene Bridged Hybrid) C18 (2.1 × 50 mm), 1.7 *μ* reversed-phase column, run in an isocratic mode, was used for chromatographic separation with the mobile phase comprising of acetonitrile/water containing 0.1% formic acid (45 : 55, *v*/*v*). Injection volumes were 5 *μ*l, the flow rate was 0.2 ml/min, and the sample was detected at 420 nm. The TQD-MS was operated under multiple reaction monitoring (MRM) mode using the electrospray ionization (ESI) technique with positive ion polarity. Data acquisition and quantification were made using Mass Lynx software version 4.1. The assay was performed using the USP reference standards of individual curcuminoids (CAS numbers: 458-37-7, 24939-17-1, and 24939-16-0).

The essential oil of turmeric was separated by hydrodistillation and characterized using gas chromatography-mass spectrometry (GC-MS). The major components present in the essential oil were characterized by Shimadzu GCMS-QP 2010 Ultra with EI source, coupled to Shimadzu Gas chromatograph GC-2010 equipped with RXI-5SI MS capillary column (30 m × 0.25 mm; film thickness 0.25 *μ*m). To begin with, the oven was programmed with an initial temperature of 80°C, which was sustained for 2 min, and the temperature was raised at a rate of 4°C/min until it reached a temperature of 240°C, and then maintained at this temperature for 5 min. The injection port temperature was ensured to be at 250°C, the flow rate of helium was 1.2 ml/min, and the detection voltage was 0.2 kV. Injection of the sample was done in split mode as 12 : 1, and the mass spectral scan range was fixed at 40-450 (m/z). Mass spectral data from the NIST11 library served as a reference to identify compounds in the sample.

### 2.3. Animals and Treatment

The selected animals were housed in cages and maintained in a room at a temperature of 22 ± 2°C and on a 12 : 12 h dark-light cycle. Food and water were provided ad libitum. The study was conducted as per the framework of CPCSEA (Committee for the Purpose of Control and Supervision of Experiments on Animals) guidelines after getting approval from the institutional animal ethics committee (NCOP/IAEC/Approved/70/2014 dated 15/3/2014).

Swiss albino mice weighing 22-28 g of both sexes were selected (*n* = 6). Pharmacokinetics and organ distribution were ascertained for turmeric extract (TE) and turmeric extract-essential oil combination (TE+EO). Aluminum chloride was used in a dose of 40 mg/kg/day and administered by the intraperitoneal (i.p.) route [15]. The neurotoxicity study was done with the following groups: (1) vehicle control [0.3% carboxymethyl cellulose (CMC)], (2) positive control (AlCl_3_-treated; 40 mg/kg, i.p.), (3) TE+EO (25 mg/kg, oral)+AlCl_3_-treated (40 mg/kg, i.p.), and (4) TE+EO (50 mg/kg, oral)+AlCl_3_-treated (40 mg/kg, i.p.). TE+EO was suspended in 0.3% CMC and fed to mice orally for 45 days. The dose of TE+EO was decided based on a previous study wherein it was administered at a dose of 50 mg/kg body weight [16]. Aluminum chloride was dissolved in distilled water and injected intraperitoneally for the same period.

### 2.4. Behavioral Studies

#### 2.4.1. Morris Water Maze Test

To assess spatial learning and memory, a water maze that consisted of a black circular water pool filled with water (25°C) to a depth of 20 cm was used. Four equally distant points along the pool's perimeter served as the starting locations where a small platform (19 cm height) was placed in the center of one of the quadrants [17]. The platform was visible and kept in the same position during the training days, and the animal had to swim to find the hidden platform. External spatial visual cues remained unchanged throughout the study and could be used by the mice for spatial orientation. The water maze task was carried out for each mouse on three consecutive days with four consecutive daily training trials. Each trial had a maximum time of 90 sec and a trial interval of around 30 seconds. For each trial, mice were placed in water at one of the four starting positions. During test trials, mice were placed in the pool at the same starting point, with their heads facing the wall, and they had to swim until it reached the platform. After climbing onto the platform, they could occupy the platform for 20 s before initiating the next trial. If the mice failed to locate the escape platform within a cut-off time of 90 s, it was gently placed on the platform and allowed to remain there for the same amount of time. Four days later, the time a mouse takes to reach the submerged platform (escape latency in seconds) was measured.

#### 2.4.2. Elevated Plus Maze Test

The elevated plus maze consisted of two opposite black open arms (50 × 10 cm), crossed with two closed walls of the same dimensions with 40 cm high walls. The arms were connected to a central square of dimensions 10 × 10 cm, and the maze was elevated 50 cm above the ground. Mice were placed individually at one end of the open arm facing away from the central square. The time the animals take to move from the open arm to the closed arm was recorded on day 42. After twenty-four hours, the time of first and second retentions was assessed to determine the acquisition and retention memory.

### 2.5. Analysis of Curcumin, Derivatives, and Metabolites

Blood samples were collected from each mouse at 1, 2, 3, 4, and 6 h time points via retroorbital plexus into K3EDTA-coated tubes, and the separated plasma was stored at -80°C until analysis. After the 6th hour of blood collection, mice were sacrificed by cervical dislocation; the brain was harvested and stored at -80°C for further studies. Plasma levels of curcuminoids and its metabolites were determined by liquid-liquid extraction with ethyl acetate/methanol [18] using salbutamol 200 ng/ml as the internal standard [19]. The brain samples were homogenized in Ringer's HEPES buffer (RHB) and then extracted with ethyl acetate. The UPLC system with ESCI-MS/MS (Waters, USA) was used for analysis. The chromatographic separation was achieved by a C18 column (120Ao, 1.0 × 100 mm, 5.0 *μ*m); analytes were eluted using acetonitrile and 0.1% formic acid in water (50 : 50, *v*/*v*). The primary stock solution was prepared for each standard, and appropriate dilutions were done to make working stock solutions. Calibration standards and control samples were prepared by spiking plasma with the appropriate working mix solution of curcumin derivatives and metabolites. The analysis of curcumin from the plasma [18] and brain [19] was partially validated before analysis. The detection limit was 0.01 ng/ml, and quantification limit was established at 0.1 ng/ml. The concentration of compounds was linear within a range of 50% to 150% of the sample concentration, and the *y*-intercept did not show a significant deviation from zero. The accuracy and precision were determined based on 80-120% of sample concentration. The extraction recovery was around 85% for curcumin, its derivatives, and 87% for metabolites. Method selectivity and sample stability during the storage and analytical process were appropriate. The repeatability was established over 80-120% of sample concentration and confirmed with three quality control samples with six replicates.

### 2.6. Biochemical Assessments

After mice were sacrificed, the hippocampus was immediately removed, and the brain homogenate was prepared. Lipid peroxidation, total protein, glutathione (GSH), superoxide dismutase (SOD), catalase (CAT), and acetylcholinesterase (AchE) levels were assessed. Lipid peroxidation was assessed by the method of Högberg et al. [20], and the results were expressed as nM malondialdehyde (MDA) released/mg of protein. The total protein content of the homogenates was determined by the method of Lowry et al. [21]. Glutathione concentration was calculated using the method described by Moron et al. and expressed as mmol/mg protein [22]. Superoxide dismutase was determined following the procedures described by Misra and Fridovich, and the SOD activity was expressed as U/mg protein [23]. The CAT activity was measured by assessing the degradation of hydrogen peroxide (H_2_O_2_) described by Aebi (1984) and reported as U/mg protein [24]. Acetylcholinesterase (AchE) levels were determined by the method of Ellman et al. (1961) method [25].

### 2.7. Histopathology

A portion of the hippocampus was fixed in formalin buffer (10%) for 24 hours, and then washed in saline and dehydrated using serial dilutions of alcohol. Specimens were cleared in xylene, embedded in paraffin, and sectioned at five microns using a microtome. The tissue sections were collected on a glass slide, deparaffinized, stained with hematoxylin and eosin, and observed under a light microscope.

### 2.8. Statistical Analysis

Pharmacokinetic analysis was conducted using the PKNCA package in the statistical tool R 4.0. Data of pharmacokinetic analysis, behavioral studies, and biochemical assessment were shown as the mean ± standard error of the mean (SEM) and were compared by one-way analysis of variance (ANOVA) using SPSS version 21. *p* < 0.05 was considered as statistically significant.

## 3. Results

### 3.1. Phytochemical Analysis

The calibration curves of curcumin, dimethoxycurcumin, and bisdemethoxycurcumin were linear over the concentration range of 1–1000 ppb. The major product ions in the positive mode were at m/z 369.2, 339.2, and 309.2, respectively (Figure 1). Curcumin, demethoxy curcumin, and bisdemethoxycurcumin were eluted at 3.39, 3.10, and 2.82 min, respectively. TE contained 95% total curcuminoids, and TE+EO contained 89.86% total curcuminoids and 7% essential oil of turmeric. GC-MS confirmed the presence of Ar-turmerone at retention time 33.337 min. Ar-turmerone was the major component present in the essential oil with a percentage area of 48.48% (Figure 2).

### 3.2. Morris Water Maze Test

The experimental mice assigned to the control group learn to locate the hidden platform using visual cues. There was a significant increase (*p* < 0.05) in escape latency time in Al-treated mice compared to the control animals. A low dose, as well as a high dose, of TE+EO significantly reduced the time taken by the animals to find the platform compared with the aluminum-treated group (*p* < 0.05). The latency time for the TE+EO (50 mg/kg) group was almost identical to the vehicle control group (Table 1).

### 3.3. Elevated Plus Maze Test

The first and second retention times representing the time taken to move from the open arms to the enclosed arms of the maze were significantly increased in mice treated with Al (*p* < 0.05) compared to the vehicle control. A statistically significant difference in the first and second retention times was observed with TE+EO (25 mg/kg and 50 mg/kg) when compared with the aluminum-treated groups (*p* < 0.05). Treatment of mice with 50 mg/kg TE+EO significantly reversed Al-induced changes, as evidenced by a decrease in the first and second retention times (Table 1).

### 3.4. Biochemical Parameters in the Brain

After 45 days of Al administration, a significant reduction (*p* < 0.05) in total protein level and AchE activity in the mouse brain was observed compared with vehicle control. Simultaneous oral administration of TE+EO restored the total protein level and AchE level, and the change was significant compared with Al-treated control mice (*p* < 0.05). Similarly, chronic administration of Al significantly elevated lipid peroxide (MDA) levels and decreased the levels of GSH and the activity of CAT when compared to control animals (*p* < 0.05). Coadministration of 25 and 50 mg/kg of TE+EO with Al significantly reduced lipid peroxide levels and was comparable with the vehicle control group. Aluminum exposure increased the activity of SOD significantly (*p* < 0.05) in comparison to vehicle control group animals, and coadministration of TE+EO significantly reduced the effect of aluminum exposure. A higher dose of TE+EO normalized GSH and CAT activity and was comparable with the vehicle control group (Table 1 and Figure 3).

### 3.5. Histopathology of the Brain

Chronic Al-treated animals showed a marked deterioration in the hippocampal region as visualized by extensive cytoplasmic vacuolation and damage to the pyramidal cells compared with vehicle-treated animals (Figure 4). Treatment with TE+EO alone exhibited a similar effect as the control group. TE+EO (25 and 50 mg/kg) minimized damage to pyramidal cells and vacuolization induced by Al treatment.

### 3.6. Pharmacokinetic Study

This is the first study to measure the efficacy, pharmacokinetics, and tissue distribution of turmeric extracts in an Al-induced neurotoxicity model to understand if plasma bioavailability and brain distribution of curcumin are related to its neuroprotective effects. The plasma concentration-time profiles of curcumin, curcuminoids, conjugated metabolites, and hydrogenated metabolites are presented in Table 2, Figure 5, and Figure 6. The curcuminoids identified were curcumin, demethoxycurcumin (DMC), and bisdemethoxycurcumin (BDMC). The conjugated metabolites included curcumin glucuronide (CG) and curcumin sulfate (CS). Also, hydrogenated or reduced metabolites included tetrahydrocurcumin (THC) and hexahydrocurcumin (HHC). TE+EO showed a significant increase in all analyte levels in the plasma and brain compared to TE alone.

TE+EO-25 provided 37.68-fold, 45.85-fold, 8.22-fold, and 9.45-fold higher AUC (0 − *α*) of curcumin, curcuminoids, conjugate metabolites, and hydrogenated metabolites, respectively, compared to TE-25. TE+EO-50 provided 121.86-fold, 114.29-fold, 10.38-fold, and 12-fold higher AUC (0 − *α*) of curcumin, curcuminoids, conjugate metabolites, and hydrogenated metabolites, respectively, compared to TE-50. TE+EO-50 provided 4.23-fold, 4.14-fold, 1.51-fold, and 1.69-fold higher AUC (0 − *α*) of curcumin, curcuminoids, conjugate metabolites, and hydrogenated metabolites, respectively, compared to TE+EO-25. TE-50 provided 1.31-fold, 1.66-fold, 1.19-fold, and 1.33-fold higher AUC (0 − *α*) of curcumin, curcuminoids, conjugate metabolites, and hydrogenated metabolites, respectively, compared to TE-25.

The curcuminoids to conjugate metabolite AUC (0 − *α*) ratio of TE+EO-25 and TE+EO-50, respectively, were 1 : 4.2 : 1 : 1.6, while the similar ratios of TE-25 and TE-50, respectively, are 1 : 23.6 and 1 : 16.9. These results clearly illustrate the characteristic drawbacks of the oral administration of turmeric extract. TE+EO (50 mg/kg) displayed the optimal pharmacokinetic profile of curcuminoids with *C*max of 99.74 ± 4.83 ng/gm and AUC 0-6 h of 439.64 ± 26.88 h ng/gm.

Curcumin, curcuminoids, and metabolites of curcumin distributed in whole-brain homogenate were estimated at 6 h for the TE+EO and TE groups. Table 2 shows the distribution of curcumin and its metabolites present in the brain fractions. TE+EO-25 provided 11.01-fold, 13.85-fold, 0.46-fold, and 7.94-fold higher concentrations of curcumin, curcuminoids, conjugate metabolites, and hydrogenated metabolites, respectively, in the brain homogenate compared to TE-25. TE+EO-50 provided 13.71-fold, 11.69-fold, 0.63-fold, and 3.92-fold concentrations of curcumin, curcuminoids, conjugate metabolites, and hydrogenated metabolites, respectively, in the brain homogenate compared to TE-50. TE+EO-50 provided 2.13-fold, 2.21-fold, 2.96-fold, and 1.39-fold higher concentrations of curcumin, curcuminoids, conjugate metabolites, and hydrogenated metabolites, respectively, in the brain homogenate compared to TE+EO-25. TE-50 provided 1.71-fold, 2.62-fold, 2.15-fold, and 2.82-fold higher concentrations of curcumin, curcuminoids, conjugate metabolites, and hydrogenated metabolites, respectively, in brain homogenate compared to TE-25.

The curcuminoids to conjugate metabolite concentration ratio of TE+EO-25 and TE+EO-50, respectively, in brain homogenate, were 374.4 : 1 and 279.6 : 1, and those of TE-25 and TE-50, respectively, were 12.5 : 1 and 15.2 : 1. The results showed that free curcumin and curcuminoids from TE+EO were chiefly distributed in the brain tissue and significantly higher than that of TE.

## 4. Discussion

The present study demonstrated the potential of formulated turmeric extract and essential oil combination in attenuating Al-induced cognitive deficits and toxicity in mice. Curcumin targets pathways involved in the pathophysiology of neurodegenerative diseases such as the *β*-amyloid cascade, tau phosphorylation, neuroinflammation, and oxidative stress. These findings suggest that curcumin can be considered as a therapeutic option to limit neuroinflammation in neurodegenerative disorders. However, low bioavailability and permeability across the blood-brain barrier limits the therapeutic potential of curcumin. The delivery of free curcumin to target tissues can be achieved by improving the bioavailability in the plasma and brain to obtain the adequate therapeutic outcomes.

Curcuminoids are the phenolic yellowish pigments of turmeric present as curcumin (CUR), demethoxycurcumin (DMC), and bisdemethoxycurcumin (BDMC). Orally administered curcuminoids are absorbed in the gut, carried to the liver, and are rapidly metabolized. Curcuminoids are metabolized in the liver and the intestinal mucosa to tetrahydrocurcumin (THC) and hexahydrocurcumin (HHC) by phase I metabolism. Curcuminoids and their reductive products are extensively conjugated with glucuronic acid and sulfate by phase II metabolism and form curcumin glucuronide and curcumin sulfate [26]. It is perceived that curcumin concentration in the brain was deficient due to the low systemic absorption and poor transport across the blood-brain barrier [27, 28]. Thus, the remedial measure was to enhance the dose of curcumin to elicit a neuroprotective response. However, the use of TE+EO achieved significantly higher (*p* < 0.05) levels of curcumin in the brain compared to TE alone. This is probably the first study reporting the simultaneous quantification of curcumin, curcuminoids, and primary and secondary metabolites in the brain and plasma after oral administration. The enhancement of brain and plasma bioavailability even at low dose (HED 142 mg in 70 kg adult) was due to the presence of turmerones in TE+EO, which acts as inhibitors of the p-glycoprotein pathway, the significant bottleneck in curcumin absorption [29]. The oral intake of bioactive turmeric extract could deliver sustained levels of free curcumin and curcuminoids. Moreover, the significantly high mean residence time (MRT), area under the curve (AUC), and *t*-half (*p* < 0.05) with TE+EO explain their neuroprotective effects. The increased bioavailability is in line with the study done on curcumin alone vs. curcuminoids with turmerones, which showed a sixfold increase in the bioavailability with the latter [30], and another study proposing the use of turmerones along with curcumin instead of curcumin alone for better therapeutic utility [29]. The administration of TE+EO also led to higher levels of THC and HHC in blood plasma and the brain, which also has pharmacological activity [31, 32]. Free curcumin was predominantly higher in the brain than its metabolites, while metabolites were higher in the blood. The low levels of curcumin and metabolites in the brain in the TE group also reflected its poor pharmacokinetic profile.

Chronic Al exposure leads to its accumulation in the brain as it is slowly removed, owing to its long half-life. Aluminum can suppress or interfere with the expression of antioxidants [33–35]. We found that Al treatment caused elevation in lipid peroxide levels in brain tissue and significant memory decline in animals. This implies an alteration in homeostasis and damage to neuronal biomolecules [36], leading to dysfunction. In the current study, although lipid hydroperoxides and lipid peroxidation have increased in the tissues, there was a corresponding increase in the protective antioxidant enzymes denoting that brain tissue could quench increased ROS and oxidative stress with TE+EO. GSH depletion can enhance oxidative stress and may also increase the levels of excitotoxic molecules. GSH functions as a free radical scavenger, particularly effective against the OH radical. The ability of GSH to nonenzymatically scavenge both singlet oxygen and OH provides the first line of antioxidant defense. SOD is an antioxidant enzyme which gets activated when there is oxidative stress and ROS formation, in case of our study due to Al. GSH reacts nonenzymatically with ROS. Oxidative stress increases the activity of GSHPx, which catalyzes the reduction of hydrogen peroxide (H_2_O_2_) by oxidizing GSH, leading to its depletion. Conditions of oxidative stress, such as GSH depletion and increased H_2_O_2_ steady-state levels, may favor the catalase pathway for H_2_O_2_ removal. Aluminum in the presence of transition metals like Fe causes lipid peroxidation generating H_2_O_2_ which is quenched by GSHPx and catalase. Furthermore, compromised antioxidant enzymes would undoubtedly have an unfavorable impact on the central nervous system. The findings of the current study indicate that the use of 50 mg/kg TE+EO counterbalances aluminum-induced free radical-mediated injury of neural tissue. Curcumin, a quencher of ROS, modulates oxidative stress by normalizing SOD enzyme activity and catalase levels plausibly by forming a ligand with Fe. Our study results show that GSH levels decreased in response to Al, indicating its role in removing H_2_O_2_. On administering TE+EO, the levels of GSH were elevated to normal due to the inhibition of lipid peroxidation. The results of the current study are supported by the findings of AlBasher et al., 2020, which show that curcumin along with resveratrol protects against fipronil-induced oxidative stress in the brain [37]. Also, curcumin along with diallyl sulfide boosts the cellular antioxidant status [38]. The essential oil of turmeric contains terpenes which facilitate the passage of curcumin in the brain as observed through our pharmacokinetic findings. Also, the constituents present in the essential oil might synergize with curcumin in displaying its antioxidant effects. Ar-turmerone, an important constituent present in the essential oil, is reported to have antioxidant action [39].

In vitro studies show that aluminum significantly accelerates iron-mediated lipid peroxidation under acidic and neutral conditions. The discovery of elevated levels of lipid hydroperoxide in the brain tissues of mice substantiates the higher phase of lipid peroxidation and oxidative stress following exposure to Al. Administration of TE+EO in a higher dose reversed the deleterious effect of Al, resulting in a significant increase in the levels of GSH, CAT, SOD, and total proteins.

Aluminum impacts the hippocampus [40] and complexes with acetylcholine [41], resulting in irreversible memory deficits [42, 43]. The potential of TE+EO in protecting neural tissues is further proved through the response observed in behavioral models. Aluminum increases latency to find the platform or transit from the open to the closed arms, implying the poor functioning of neurons involved in learning and memory. Aluminum-exposed animals exhibited cognitive impairment, which was significantly reversed with the use of 50 mg/kg of TE+EO as evidenced through the Morris water maze and elevated plus maze task; however, 25 mg/kg exhibited a significant response in improving spatial memory but did not elicit improvement in transfer latency with the elevated plus maze. The role of TE+EO in improving cognitive function could mechanistically be explained by its protection of biomembranes owing to its activation of antioxidant systems and reduced formation of free radicals.

Learning and memory are correlated mainly with the cholinergic system and the availability of acetylcholine. Acetylcholinesterase plays a vital part in the functioning of nerves, and severe physioIogica1 damage arises from its blockage. When the action of acetylcholinesterase is blocked, acetylcholine accumulates, leading to endogenous poisoning. Our study results show that the levels of AChE decreased in response to Al, and TE+EO elevated it to the normal levels. Only 50 mg/kg of TE+EO was effective in increasing the levels of acetylcholinesterase, and the same dose also improved memory assessed through the behavioral models confirming the efficacy of TE+EO at this dose level. Moreover, 50 mg/kg of TE+EO protected the hippocampus from Al-induced damage plausibly by improving the defense system, suppressing lipid peroxide levels, and increasing the availability of curcuminoids in the presence of turmerones in the formulation. Furthermore, the expression of transcription factors could be indirectly impacted, shielding neuronal structures against peroxidative damage. Imbalances in the oxidant-antioxidant status can be a trigger for inflammation. TE+EO might prevent inflammatory damage of neurons. The anti-inflammatory effects of TE+EO have been reported in colitis induced by dextran sulfate [44].

Histopathological changes of the hippocampus in Al-treated animals have further attested to the biochemical and behavioral results characterized by damage to pyramidal cells, which are in line with other studies [2, 45]. CA3 pyramidal neurons play an important role in conveying neural information to the CA1 neurons; hence, damage to this field could affect recall of memories recently learned. We observed that the 50 mg/kg of TE+EO protects the hippocampal neurons, enabling the circuit to work efficiently resulting in a favorable behavioral outcome.

## 5. Conclusion

Turmeric extract and essential oil combination works in unison to reverse the effects produced by the chronic exposure of Al, firstly, by enabling more plasma bioavailability and access of curcuminoids into the brain and, secondly, by upregulating the expression of antioxidants, thereby minimizing microglia activation and subsequent neuronal damage. The observed effect of TE+EO could be linked with its ability to cross the blood-brain barrier, bind to redox metal ions, and neutralize free radicals. This makes TE+EO a promising therapeutic option for prophylaxis and treatment of neurodegenerative diseases as it could substantially reduce neuroinflammation and oxidative stress and improve memory in mice exposed to aluminum.

## Figures and Tables

**Figure 1:** The LC-MS/MS total ion chromatogram of TE+EO.

**Figure 2:** Gas chromatography-mass spectrum (GC-MS) of essential oil of turmeric.

**Figure 3:** Influence on biomarkers of the mouse brain homogenate of the aluminum and TE+EO groups when compared to the control group.

**Figure 4:** H&E-stained slides of the hippocampal CA1 area in mice exposed to aluminum and simultaneously treated with TE+EO. (a) Vehicle control showing normal cells. (b) Aluminum chloride- (AlCl_3_-) treated showing shrunken, vacuolated, and degenerated neurons. (c) AlCl_3_+TE+EO-25 showing improvement. (d) AlCl_3_+TE+EO-50 resulted in reduction in vacuolization.

**Figure 5:** Plasma concentration-time curve of curcumin after administration of TE+EO (25 and 50 mg/kg) and TE (25 and 50 mg/kg).

**Figure 6:** Mean of AUC (0 to *α*) of curcuminoids and its metabolites from the TE and TE+EO groups.

**Table 1:** Impact of turmeric extract and essential oil combination on cognitive performance and biochemical parameters in aluminum chloride-treated mice.

Treatment	Morris water maze	Elevated plus maze		Total proteins (mg/g tissue)	MDA (nM released/mg protein)	GSH (*μ*M/mg tissue)	SOD (U/mg protein)	CAT (U/mg protein)	AchE (nM/mg protein)
	Escape latency (sec)	1st retention (sec)	2nd retention (sec)						
Control (vehicle)	33.17 ± 1.30^bc^	35.17 ± 1.38^bc^	15.67 ± 0.67^∗^^bc^	72.76 ± 1.78^bcd^	45.57 ± 2.07^b^	309.56 ± 6.69^bc^	0.58 ± 0.04bc^d^	42.72 ± 1.76^b^	3.82 ± 0.09^bcd^
Untreated control (AlCl_3_)	63.00 ± 1.59^acd^	64.17 ± 3.89^acd^	59.83 ± 2.65^acd^	35.37 ± 0.81^acd^	97.33 ± 2.50^acd^	103.91 ± 5.09^acd^	0.89 ± 0.02^acd^	28.66 ± 3.11^ad^	0.34 ± 0.05^acd^
AlCl_3_+TE+EO-25	45.00 ± 2.38^ab^	52.00 ± 0.86^abd^	33.00 ± 0.97^∗^^abd^	58.17 ± 2.48^ab^	56.23 ± 3.64^b^	246.93 ± 10.96^abd^	0.77 ± 0.03^ab^	37.63 ± 3.57	1.95 ± 0.13^abd^
AlCl_3_+TE+EO-50	38.17 ± 1.92^b^	35.33 ± 0.76^bc^	19.67 ± 0.67^∗^^bc^	60.61 ± 1.80^ab^	54.72 ± 2.98^b^	287.39 ± 5.65^bc^	0.69 ± 0.02^ab^	41.92 ± 1.92^b^	2.83 ± 0.22^abc^

Values are expressed as the mean ± standard error of the mean. ^a^*p* < 0.05 compared with the control. ^b^*p* < 0.05 compared with untreated control (AlCl_3_). ^c^*p* < 0.05 compared with the AlCl_3_+TE+EO-treated group (25 mg/kg); ^d^*p* < 0.05 compared with the AlCl_3_+TE+EO-treated group (50 mg/kg). ^∗^*p* < 0.05 comparing second retention with first retention by paired *t*-test. AlCl_3_: aluminum chloride; TE+EO: turmeric extract and essential oil combination.

**Table 2:** Pharmacokinetic parameters of curcumin, curcuminoids, and metabolites and its concentration in brain tissue.

Parameters	Group	Curcumin	Curcuminoids (curcumin+DMC+BDMC)	Conjugate metabolites (CG+CS)	Hydrogenated metabolites (HHC+THC)
		Mean ± SEM	Mean ± SEM	Mean ± SEM	Mean ± SEM
*t*1/2	TE+EO-25	3.31 ± 0.51^b^	3.20 ± 0.46^bcd^	1.91 ± 0.16^cd^	1.68 ± 0.14^d^
	TE+EO-50	8.04 ± 1.70^acd^	6.01 ± 1.17^acd^	1.56 ± 0.17^cd^	1.68 ± 0.16^d^
	TE-25	2.05 ± 0.43^b^	0.39 ± 0.03^ab^	0.86 ± 0.06^ab^	1.26 ± 0.13^d^
	TE-50	2.06 ± 0.52^b^	0.52 ± 0.05^ab^	0.87 ± 0.05^ab^	0.40 ± 0.02^abc^
*T*max	TE+EO-25	3.50 ± 0.22^bcd^	3.50 ± 0.22^bcd^	1.00 ± 0.00	1.83 ± 0.17
	TE+EO-50	2.17 ± 0.17^a^	2.33 ± 0.21^a^	1.00 ± 0.00	1.83 ± 0.17
	TE-25	1.83 ± 0.17^a^	2.00 ± 0.00^a^	2.00 ± 0.00	2.17 ± 0.17
	TE-50	2.33 ± 0.21^a^	2.17 ± 0.17^a^	2.00 ± 0.00	2.17 ± 0.17
*C*max	TE+EO-25	32.00 ± 2.22^bcd^	34.23 ± 2.19^bcd^	297.91 ± 9.86^bcd^	16.75 ± 0.74^bcd^
	TE+EO-50	79.60 ± 6.91^acd^	99.74 ± 4.83^acd^	471.77 ± 12.85^acd^	28.11 ± 1.20^acd^
	TE-25	1.27 ± 0.20^ab^	1.41 ± 0.19^ab^	47.81 ± 5.88^ab^	2.43 ± 0.26^ab^
	TE-50	1.59 ± 0.43^ab^	2.48 ± 0.35^ab^	56.63 ± 3.73^ab^	3.45 ± 0.38^ab^
AUC 0-*t*	TE+EO-25	141.86 ± 9.40^bcd^	152.26 ± 9.32^bcd^	904.17 ± 43.70^bcd^	60.36 ± 1.92^bcd^
	TE+EO-50	357.24 ± 32.51^acd^	439.64 ± 26.88^acd^	1429.96 ± 35.44^acd^	101.63 ± 3.24^acd^
	TE-25	4.72 ± 0.81^ab^	5.37 ± 0.82^ab^	124.98 ± 15.88^ab^	6.53 ± 0.29^ab^
	TE-50	6.59 ± 1.81^ab^	8.90 ± 1.93^ab^	149.84 ± 8.61^ab^	9.81 ± 0.46^ab^
AUC 0-inf	TE+EO-25	234.34 ± 22.21^b^	247.11 ± 23.12^b^	1045.76 ± 54.11^bcd^	70.01 ± 3.12^bcd^
	TE+EO-50	991.90 ± 187.40^acd^	1024.00 ± 177.14^acd^	1581.53 ± 51.15^acd^	118.24 ± 5.84^acd^
	TE-25	6.22 ± 1.10^b^	5.39 ± 0.82^b^	127.18 ± 16.21^ab^	7.41 ± 0.41^ab^
	TE-50	8.14 ± 1.70^b^	8.96 ± 1.94^b^	152.30 ± 8.87^ab^	9.85 ± 0.46^ab^
MRT	TE+EO-25	6.21 ± 0.68^b^	6.06 ± 0.60^b^	3.32 ± 0.16^cd^	3.46 ± 0.14^d^
	TE+EO-50	12.43 ± 2.47^acd^	9.65 ± 1.67^acd^	2.99 ± 0.15	3.47 ± 0.18^d^
	TE-25	3.96 ± 0.50^b^	2.69 ± 0.04^b^	2.69 ± 0.03^a^	3.07 ± 0.15
	TE-50	4.54 ± 0.75^b^	2.79 ± 0.07^b^	2.62 ± 0.04^a^	2.73 ± 0.04^ab^
Concentration in the brain	TE+EO-25	65.75 ± 4.39^bcd^	89.86 ± 5.51^bcd^	0.24 ± 0.16^d^	1.35 ± 0.14^c^
	TE+EO-50	140.07 ± 8.19^acd^	198.53 ± 10.12^acd^	0.71 ± 0.31	1.88 ± 0.52^cd^
	TE-25	5.97 ± 0.94^ab^	6.49 ± 0.93^ab^	0.52 ± 0.09	0.17 ± 0.10^ab^
	TE-50	10.22 ± 0.81^ab^	16.98 ± 1.20^ab^	1.12 ± 0.16^a^	0.48 ± 0.11^b^

*t*1/2: terminal phase half-life; *T*max: time to maximum plasma concentration; *C*max: maximum concentration; AUC (0-6 h): area under the curve up to 6 h; AUC (0-∞): AUC up to infinite time; MRT: mean residence time. ^a^*p* < 0.05 when compared to TE+EO-25. ^b^*p* < 0.05 when compared to TE+EO-50. ^c^*p* < 0.05 when compared to TE-25. ^d^*p* < 0.05 when compared to TE-50.

## Data Availability

The datasets used and/or analysed during the current study are available from the corresponding author on reasonable request.
